# Reduced interleukin-38 in non-small cell lung cancer is associated with tumour progression

This article has been retracted.

**DOI:** 10.1098/rsob.180132

**Published:** 2018-10-31

**Authors:** Feng Wang, Weihua Zhang, Tianfeng Wu, Heying Chu

**Affiliations:** 1 Department of Respiration, The 1st Hospital of Shangqiu, Shangqiu 476100, People's Republic of China; 2 Department of Cancer, The 1st Hospital of Shangqiu, Shangqiu 476100, People's Republic of China; 3 Department of Respiration, The First Affiliated Hospital of Zhengzhou University, Zhengzhou 450002, People's Republic of China

**Keywords:** IL-38, non-small cell lung cancer, interleukin-38

## Abstract

Lung cancer continues to be the leading cause of cancer-related deaths worldwide due to its high incidence, malignant behaviour and lack of major advancements in treatment strategy. The occurrence and development of lung cancer is closely related to inflammation. Thus, we conducted the present study to investigate the effects of IL-38 (interleukin-38), a newly identified anti-inflammatory factor, on non-small cell lung cancer (NSCLC), which accounts for about 85% of all lung cancers. We first evaluated the IL-38 expression in 384 pairs of NSCLC samples and their adjacent normal mucosa by real-time PCR, ELISA (enzyme-linked immunoassay) and tissue microarrays. Then the role of IL-38 on patient survival rates, cancer progression and their sensitivity to chemotherapy drugs was assessed. IL-38 was barely expressed in the NSCLC tissues but highly expressed in the adjacent normal tissues. The downregulation of IL-38 was significantly correlated with the results of the American Joint Committee on Cancer stage and degree of differentiation, and it was also shown to be an independent prognostic indicator of disease-free survival and overall survival for patients with NSCLC. Overexpression of IL-38 in NSCLC cells suppressed cell migration, invasion, proliferation and colony formation through suppressing β-catenin. IL-38 inhibited NSCLC formation in a mice model and sensitized the cancer cells to chemotherapy drugs. Our results show that IL-38 plays an inhibitory role in NSCLC development and functions as a novel prognostic indicator and a potential therapeutic target.

## 1. Introduction

Lung cancer is currently the most common cause of tumour-related mortality in the world [1–3]. There are two main subtypes of lung cancer, small-cell lung carcinoma and non-small cell lung carcinoma (NSCLC), accounting for 15% and 85% of all lung cancer, respectively [1–4]. Clinically, NSCLC is frequently diagnosed at advanced stages of disease [4]. Over half of patients diagnosed with lung cancer die within one year of diagnosis and the 5-year survival rates are around 17.8% [1–3]. Moreover, NSCLC patients are relatively insensitive to chemo- and radiotherapy [4]. Despite advances in early detection, radical surgical resection and multimodal therapeutic modalities over recent decades, the long-term survival remains poor due to the high rate of recurrence and metastasis [1].

Therefore, there is an urgent need to identify novel biomarkers that will help select the patients with high chance of lung cancer recurrence and uncover the underlying mechanisms which would provide better targets for NSCLC treatment. Dysregulated inflammatory response is related to an increased risk of chronic disease and cancers, including lung cancer [5], and pro-inflammatory cytokines play an important role in many tumour-related processes, including growth, metastasis, apoptosis and angiogenesis [6]. Interleukin-38 (IL-38) is a newly identified anti-inflammatory factor in the IL-1 ligand family [7,8]. IL-38 binds to IL-36R similarly to IL-36Ra, which can inhibit the pro-inflammatory function of IL-36 [9]. However, the role of IL-38 in NSCLC remains unknown.

Thus, we conducted the present study to investigate the effects of IL-38 on NSCLC. To address the role of IL-38 in NSCLC, we first evaluated IL-38 expression in human NSCLC tissues; then the IL-38 function was assessed *in vitro* and *in vivo* in a xenografted lung tumour model. The results indicate that IL-38 might play an important role in NSCLC progression and function as a novel prognostic indicator and a potential therapeutic target.

## 2. Methods and materials

### 2.1. Patients

A total of 384 patients with histologically verified NSCLC at the First Affiliated Hospital of Zhengzhou University, between 2005 and 2015, were enrolled in this study. The median age of the patients was 57.5 years (range 28–71 years). None of them received any preoperative anti-cancer treatment prior to sample collection. This study was approved by the local ethics committee of the First Affiliated Hospital of Zhengzhou University, and written informed consent was obtained from each patient. All 384 specimens were re-evaluated with respect to their histological types, differentiation status, smoking status and tumour TNM stages. Tumour stages were determined by TNM classification according to the 2002 International Union against Cancer guidelines. The histological diagnosis and grade of differentiation of the tumours were defined by evaluation of haematoxylin and eosin (H&E)-stained tissue sections, according to the 2004 World Health Organization guidelines for classification. Tissues were collected within 1 h after surgery. Every patient specimen included two matched pairs, namely NSCLC tissues and adjacent normal lung tissues (greater than or equal to 5 cm away from the tumour). For each specimen, half was immediately flash-frozen in liquid nitrogen and then frozen at −80°C until RNA and protein extraction was performed, and the remainder was fixed with formalin for immunohistochemistry.

### 2.2. RNA extraction and real-time polymerase chain reaction

Total RNA was extracted from samples with Trizol (Invitrogen, Carlsbad, CA) according to the manufacturer's instructions. Then the quantity and purity of RNA was determined by absorbance on a FilterMax F5 Multi-Mode Microplate Reader (Sunnyvale, CA) at 260 nm and 280 nm. Samples with ratios from 1.8 to 2.0 were accepted for reverse transcription reaction. cDNA was prepared using the iScript™ cDNA Synthesis kit (Bio-Rad, USA). β-Actin was used as an internal control. The RT-PCR amplification reaction was prepared with the SYBR Green PCR kit (Bio-Rad, USA) and performed using the 7500 fast Real-Time PCR system (Applied Biosystems, USA). PCR products were verified by melting curve analysis. Relative mRNA levels of target genes were calculated by the 2^−ΔΔct^ method.

### 2.3. Enzyme-linked immunoassay

The protein level of IL-38 was detected in tumour homogenate using a human IL-38 ELISA kit (AdipoGen AG, Liestal, Switzerland) according to the manufacturer's instructions. All samples were assayed in triplicate.

### 2.4. Western blotting

Total protein from tumour tissues and cultured cells was lysed in RIPA buffer with protease inhibitor (Beyotime, Shanghai, China). The protein was quantified using a BCA assay kit (Beyotime, Shanghai, China). A total of 20 µg of total protein was separated by 10% SDS-PAGE, transferred onto polyvinylidene fluoride membranes and then reacted with primary antibodies against IL-38 (Thermo Scientific, USA), β-catenin and β-actin (Abcam, Cambridge, UK). After being extensively washed with PBS containing 0.1% Triton X-100, the membranes were incubated with alkaline phosphatase-conjugated goat anti-rabbit antibody for 30 min at room temperature. The bands were visualized using 1-step TM NBT/BCIP reagents (Thermo Fisher Scientific, Rockford, IL) and detected by an Alpha Imager (Alpha Innotech, San Leandro, CA).

### 2.5. Tissue microarrays construction and immunohistochemistry

Formalin-fixed, paraffin-embedded samples, including primary tumours and paired normal mucosa, were analysed. Representative areas of tissue were established by microscopic review of H&E stained slides and 2.0 mm diameter cores were punched from the paraffin blocks. Two cores from each of the primary cancer and normal tissues at a distance of at least 2 cm from the tumour were arrayed. Tissue microarrays (TMAs) were created using a Tissue Microarrayer (Beecher Instruments, Sun Prairie, WI, USA). All specimens were examined by at least two pathologists to prevent bias. Tumour and normal mucosa morphology on the arrays were validated as having high accordance with that of the whole archived section.

For IL-38 immunostaining, a microwave-based antigen retrieval process was employed with EDTA buffer, pH 8.0, for 30 min. After the sections had been cooled, endogenous peroxidase was inhibited with 3% hydrogen peroxide for 10 min at room temperature. Non-specific binding was blocked with fetal calf serum for 15 min before incubation of the sections with mouse anti-human IL-38 antibody (Thermo Scientific, USA) at 4°C overnight. As a negative control, sections were incubated with normal mouse IgG. After being incubated with the primary antibodies, the sections were then incubated with horseradish peroxidase (HRP)-labelled anti-mouse IgG at 37°C for 30 min, followed by visualization with 3,3-diaminobenzidine (DAB) and counterstaining with Mayer's haematoxylin. The desired colour reaction was observed when monitored with the microscope.

Based on the intensity and extent of staining, the immunohistochemically stained slides were re-evaluated by two independent observers who were blinded to patient information. Briefly, IL-38 staining of the tumour cells was designated with an intensity score (0 (no staining), 1 (weak staining), 2 (moderate staining) and 3 (strong staining)) and an extent score (0 (no staining of cells), 1 (less than 10% of tissue stained positive), 2 (10%–50% stained positive), 3 (greater than 50% stained positive)). The intensity and extent score were then summed to give a total score ranging from 0 to 6, with a total score of 0 to 2, 3 to 4 and 5 to 6 defined as no expression, weak expression and strong expression of IL-38, respectively.

### 2.6. Recombinant human IL-38 protein expression

The *IL-38* gene (homo species) was amplified from cDNA of peripheral blood mononuclear cells. The PCR fragments were double digested with restriction endonucleases and ligated into the prokaryotic expression vector. The protein was expressed in a stable prokaryotic expression system. The plasmids of positive clones were then sequenced by the Sanger method with 100% identity with the published sequence. The induced and uninduced cultures were analysed by SDS-PAGE to identify the expression of recombinant protein. The harvested cells were resuspended in NaCl–Tris–HCl buffer, sonicated in an ice bath, and centrifuged at 12 000 r.p.m. for 30 min, and the supernatants were collected. The supernatants were added to a His Trap HP 1 ml column (GE) that had been equilibrated with NaCl–Tris–HCl buffer. Different concentrations of imidazole buffer were used to elute the recombinant protein. Collected target protein peaks were examined by SDS-PAGE electrophoresis and immunoblot analysis using anti-human IL-38 antibody. The eluted recombinant protein was dialysed in PBS at 4°C overnight. The concentration was detected by the Bradford method, and the recombinant protein was stored at −20°C.

### 2.7. Cell culture

The A549 and SK-MES-1 human NSCLC cell lines were obtained from the American Type Culture Collection (ATCC; Rockville, MD) and cultured in DMEM (GIBCO, Shanghai, China) supplemented with 10% FBS. Recombinant human IL-38 (rhIL-38) protein, with a concentration ranging from 0 to 100 ng ml^−1^ (0, 1, 10, 100 ng ml^−1^), was added to the medium after culture for 24 h.

### 2.8. Cell viability assay

Cell viability was evaluated using CCK-8 (Beyotime, Shanghai, China) according to the manufacturer's instructions. Briefly, cells were seeded into 96-well plates at 5 × 10^3^ cells per well and cultured for the indicated time points. Ten microlitres of CCK-8 solution was added into the culture medium in each well. After a 1-h incubation, OD values were read using a microplate reader (Bio-Tek Company, Winooski, VT) at a wavelength of 450 nm. Each time point was repeated in three wells and the experiment was independently performed for three times.

### 2.9. Cell apoptosis assay

Cell apoptosis was evaluated by flow cytometry using an Annexin V-FITC Apoptosis Detection Kit (KeyGen Biotech Co. Roche, Nanjing, China). Briefly, cells were seeded into 24-well plates at 1 × 10^5^ cells per well and cultured for 48 h. Then the cells were detached by trypsinization, washed twice in PBS (2000 r.p.m., 5 min; Allegra X-12R centrifuge; Beckman Coulter, USA) and resuspended in 500 µl binding buffer. A volume of 5 µl Annexin V-FITC and 5 µl propidium iodide was added and mixed gently, and the cells were stained in the dark for 10 min at room temperature. The cells were analysed immediately by flow cytometry (BD FACSCalibur, BD Bioscience, San Diego, CA) and analysed using Flowjo software (FlowJo, Ashland, OR). The experiment was repeated three times.

### 2.10. Cell migration assay

The migration of cells was detected by a wound-healing assay. Cells were cultured in six-well plates. When the cells grew to 80–90% confluence, a wound in a line across the well was made by a plastic pipette tip. The area of cell-free wound was recorded 24 h after incubation with rhIL-38 protein using an inverted microscope and analysed by NIH Image 1.55 software. Percentage wound healing was calculated as 100 × (1 − the remaining cell-free area/the area of the initial wound). All tests were performed in triplicate.

### 2.11. Transwell invasion assay

Invasive ability of cells was determined within a Transwell system. The cells (6.0 × 10^4^) were seeded onto the upper surface of the Transwell membrane and cultured at 37°C in 5% CO_2_ for 24 h, 48 h and 72 h. The number of cells that migrated to the lower surface of the membrane was counted under a microscope (200×).

### 2.12. Clonogenic assays

The cells were plated at either 1 × 10^3^ cells per well in six-well plates in standard growth media. The cells were allowed to form colonies for 10 days before being fixed and stained with 0.2% crystal violet (w:v) in 10% buffered formalin. Colony numbers were manually counted.

### 2.13. Animal study

Female 6–8 weeks old BALB/c nu/nu mice (Charles River Laboratories, Beijing, China) were housed in specific pathogen-free conditions. The study was approved by the Research Ethics Committee of the First Affiliated Hospital of Zhengzhou University. For evaluation of tumour growth *in vivo*, 1 × 10^7^ cells were suspended in 200 µl PBS and injected subcutaneously into the flank region of nude mice. Tumour growth was monitored every 2 days; tumours were measured with fine digital calipers and tumour volume was calculated by the following formula: tumour volume = 0.5 × width^2^ × length. After tumour volume reached around 60 mm^3^, the mice were subjected to IL-38 therapy. After four weeks, the mice were sacrificed, the tumours were collected and the tumour volumes were measured.

### 2.14. Production and *in vivo* delivery of adeno-associated virus

Vector construction, production and *in vivo* delivery of adeno-associated virus (AAV) were performed based on the AAV helper-free system (Agilent). The recombinant adenoviral vector pAAV-IL38 was constructed by cloning the cDNA encoding region into pAAV-ITR. The vector pAAV-GFP encoding green fluorescence protein was used as a negative control. Recombinant AAVs were produced by HEK293 cells (ATCC) transfected with pAAV-ITR vectors together with pAAV-RC and pHelper plasmids, and then purified by discontinuous iodixanol gradient centrifugation. Purified recombinant AAVs were concentrated and desalted by centrifugation through Amicon Ultra 30 K filters (Millipore). For *in vivo* delivery, recombinant AAVs equivalent to 1.0 × 10^12^ viral genome copies were delivered via the mouse tail vein.

### 2.15. Chemotherapy assay

Cells were treated with 5-fluorouracil (1.5 μM, Sigma), cisplatin (1.5 µM, Sigma) and doxorubicin (30 nM, Sigma) for 24 h. Then the cells were plated at 1 × 10^3^ well^−1^ in six-well plates. Ten days later, cells were fixed and stained with crystal violet. Dye was then solubilized with 1% SDS and OD590 was measured.

### 2.16. Statistical analysis

Data were expressed as mean (±s.e.) and analysed by a SPSS software package (SPSS Standard v. 13.0, SPSS Inc, USA). Differences between variables were assessed by the χ^2^ test. Survival analysis of patients with colorectal cancer was calculated by Kaplan–Meier analysis. A log-rank test was used to compare different survival curves. A Cox proportional hazards model was used to calculate univariate and multivariate hazard ratios for the variables. Unpaired Student's *t-*test and one-way ANOVA were used as appropriate to assess the statistical significance of difference; *p*-values less than 0.05 were considered statistically significant.

## 3. Results

### 3.1. Decreased IL-38 expression in human non-small cell lung cancer

A total of 384 cases with NSCLC were followed (table 1). All these patients had received no pre-operation chemotherapy. They were given the same radical operation and underwent the same adjuvant chemotherapy after the surgery. We first analysed IL-38 expression in 384 NSCLC specimens. The data showed that the mRNA and protein levels of IL-38 in NSCLC tissues were lower than in the paired adjacent non-cancerous tissues (figure 1*a,b*), and this was further confirmed by western blot analysis (figure 1*c*).

**Figure 1.** Lack of IL-38 expression correlated with the poor prognosis of NSCLC. (*a*) IL-38 mRNA levels in cancer tissues and adjacent normal tissues were determined by real-time PCR (*n* = 384). *p < 0.05. (*b*) IL-38 protein levels in cancer tissues and adjacent normal tissues were determined by ELISA (*n* = 384). *p < 0.05. Results are depicted as box plots; middle line indicates median; bottom of box, 25th percentile; and top of box, 75th percentile. (*c*) Representative figure for IL-38 protein levels in cancer tissues and adjacent normal tissues were determined by western blot. N: adjacent normal tissues; C: cancer tissues. (*d*) Representative figures of negative, weak or strong expression of IL-38. (*e*) Kaplan–Meier survival curves of patients with negative, weak or strong expression of IL-38.

**Table 1.** Association between clinicopathological features and IL-38 protein expression. ADC, adenocarcinoma; SCC, squamous cell carcinoma.

IL-38 expression					
	*N*	strong (*n* = 194, %)	weak (*n* = 108, %)	negative (*n* = 82, %)	*p*-value
age, years					0.393
<65	171	34.0	37.0	45.0	
≥65	213	66.0	63.0	55.0	
gender					0.521
male	181	48.4	40.7	39.1	
female	203	51.6	59.3	60.9	
T stage					0.016*
T1	6	3.2	5.5	3.0	
T2	21	16.1	13.0	5.7	
T3	173	46.9	42.5	29.1	
T4	184	33.8	39.0	62.2	
N stage					0.005*
N0	93	67.7	48.1	40.7	
N1	159	25.7	33.3	34.7	
N2	132	6.6	18.6	24.6	
M stage					0.002*
M0	267	96.8	96.3	81.3	
M1	117	3.2	3.7	18.7	
AJCC stage					0.001*
I	73	17.7	11.0	7.2	
II	118	46.8	37.0	31.9	
III	125	32.2	48.0	42.0	
IV	68	3.3	4.0	18.9	
differentiation					0.001*
high	89	66.0	50.0	32.0	
moderate	167	27.4	36.0	41.0	
low	128	6.6	14.0	27.0	
histological type					0.487
ADC	265	46.5	39.8	62.7	
SCC	119	53.5	60.2	37.3	
smoking					0.586
never	123	57.6	61.5	46.7	
smoker	261	42.4	38.5	53.3	
pleural and lymphatic invasion					0.498
positive	257	89.7	93.4	90.8	
negative	127	10.3	6.4	9.2	
vascular invasion					0.452
yes	272	96.8	92.6	91.4	
no	112	3.2	7.4	8.6	

*p < 0.05 indicates a significant association among the variables.

Immunohistochemical analysis on a tissue array showed that the lack of IL-38 expression was significantly associated with lymph node metastasis (table 1). The lack of IL-38 expression also showed a positive association with the American Joint Committee on Cancer (AJCC) stage (*p* = 0.001) and degree of differentiation (*p* = 0.001).

Patient follow-up was carried out for all patients who had undergone curative operations. Kaplan–Meier analysis with a log-rank test for overall survival (OS) and disease-free survival (DFS) was conducted to assess the predictive role of IL-38 for distant metastasis. There was a significant difference between IL-38 positive and negative groups after the surgery (figure 1*d*,*e*). Patients with IL-38 negative tumours subsequently developed more metastasis or local recurrence than those with IL-38 positive tumours (*p* < 0.01).The DFS rate was significantly lower in patients with IL-38 negative primary tumours (figure 1*e*, log-rank test, *p* < 0.001) than in patients with IL-38 positive tumours. Kaplan–Meier analysis also revealed that IL-38 expression was significantly related to OS of NSCLC patients (figure 1*e*, log-rank test, *p* < 0.001). Patients with IL-38 negative tumours had a significantly lower 5-year OS than those with IL-38 positive tumours.

Univariate analysis showed that patients with IL-38 negative NSCLC had a significantly lower DFS and OS than those with IL-38 positive tumours (table 2). In multivariate analysis with clinicopathological parameters, the lack of IL-38 expression was found to be an independent prognostic marker to predict tumour recurrence (table 3).

**Table 2.** Univariate Cox proportional hazard model for disease-free survival (DFS) and overall survival (OS). HR, hazard ratio; CI, confidence interval.

	DFS			OS		
	HR	95% CI	*p*-value	HR	95% CI	*p*-value
age, years						
<65	—			—		
≥65	1.009	0.659–1.841	0.754	0.934	0.540–1.644	0.852
AJCC stage						
I	—			—		
II	1.108	0.305–4.827	0.857	0.667	0.251–2.215	0.518
III	6.823	2.097–22.199	0.001*	3.401	1.184–9.771	0.013*
IV	49.185	12.615–191.764	<0.001*	40.074	11.257–142.648	<0.001*
differentiation						
high	—			—		
moderate	1.315	0.750–2.356	0.341	1.458	0.764–2.780	0.453
low	3.577	1.885–6.786	<0.001*	4.358	2.140–8.872	<0.001*
vascular invasion						
yes	4.901	2.469–9.731	<0.001*	4.688	2.152–9.937	<0.001*
no	—			—		
IL-38 expression						
positive	—			—		
weak	2.528	1.194–5.673	0.011*	2.147	0.882–5.126	0.152
negative	6.178	3.054–12.462	<0.001*	6.388	2.875–14.014	<0.001*

*p < 0.05 indicates a significant association among the variables.

**Table 3.** Multivariate Cox proportional hazard model for DFS and OS. HR, hazard ratio; CI, confidence interval.

	DFS			OS		
	HR	95% CI	*p*-value	HR	95% CI	*p*-value
IL-38 expression	2.726	1.919–4.161	<0.001*	2.659	1.711–4 223	<0.001*
T stage	1.751	1.129–2.541	0.005*	3.971	1.854–9.173	<0.001*
N stage	3.658	2.049–6.701	<0.001*	3.331	1.813–6.203	<0.001*
M stage	4.442	1.299–14.551	0.015*	8.041	2.403–26.815	<0.001*

*p < 0.05 indicates a significant association among the variables.

Taken together, these results suggested that the decrease in intratumoural IL-38 expression might be associated with NSCLC progression and poor clinical outcome in human NSCLC.

### 3.2. IL-38 suppresses non-small cell lung cancer in a dose-dependent manner

To further investigate the role of IL-38 in NSCLC development, cell migration, invasion, apoptosis, proliferation and cancer stem cells were analysed in two human NSCLC cell lines, A549 and SK-MES-1, after the administration of various concentrations of rhIL-38 (recombinant human IL-38). The expression of the IL-38 receptor IL-36R in NSCLC was confirmed by western blot (figure 2*a*). IL-38 inhibited the migration and invasion of A549 and SK-MES-1 cells in a dose-dependent manner (figure 2*b*,*c*). Additionally, IL-38 promoted the apoptosis of A549 and SK-MES-1 cells in a dose-dependent manner (figure 2*d*). Moreover, IL-38 dampened the proliferation of A549 and SK-MES-1 cells (figure 2*e*). Furthermore, their clone formation capability was also reduced by IL-38 (figure 2*f*). And this was further confirmed using the freshly isolated NSCLC cells (electronic supplementary material, figure S1).

**Figure 2.** IL-38 suppresses NSCLC in a dose-dependent manner. (*a*) Western blot showed the expression of IL-36R in A549 and SK-MES-1 cells. (*b*) Wound healing assay of A549 and SK-MES-1 cells with different concentrations of rhIL-38 protein (0, 1, 10, 100 ng ml^−1^). *n* = 3. *p < 0.05. (*c*) Cell invasion assay of A549 and SK-MES-1 cells with different concentrations of rhIL-38 protein (0, 1, 10, 100 ng ml^−1^). *n* = 3. *p < 0.05. (*d*) Analysis of NSCLC cell apoptosis following treatment of rhIL-38. A549 and SK-MES-1 cells were treated at the indicated doses, harvested and stained with Annexin V-FITC and 7-AAD. Annexin V-FITC-positive apoptotic cells were determined by flow cytometry. *n* = 3. *p < 0.05. (*e*) The survival rates of A549 and SK-MES-1 cells treated with different concentrations of rhIL-38 (0, 1, 10, 100 ng ml^−1^) were analysed. *n* = 3. *p < 0.05. (*f*) The clone formation number of A549 and SK-MES-1 cells treated with different concentrations of rhIL-38 (0, 1, 10, 100 ng ml^−1^) were analysed. *n* = 3. *p < 0.05.

These results indicated that an appropriate concentration of IL-38 was efficient at inhibiting the migration, invasion and proliferation, and accelerating the apoptosis of NSCLC cells. Furthermore, IL-38 could reduce the number of cancer stem cells.

### 3.3. IL-38 inhibits β-catenin expression in non-small cell lung cancer cells

We further investigated the underlying mechanism of anti-tumour effects of IL-38 in NSCLC cells. The expressions of β-catenin in A549 and SK-MES-1 cells were analysed after treatment with 100 ng ml^−1^ rhIL-38 for 24 h, because of the important role of β-catenin in NSCLC development [10]. The mRNA and protein levels of β-catenin were suppressed by IL-38 in these two cell lines (figure 3*a*,*b*). To further confirm the correlation between IL-38 and the β-catenin signalling pathway, we transfected the A549 and SK-MES-1 cells with plasmids overexpressing IL-38, β-catenin or both together. Compared with the control group, the effects of IL-38 on cell migration, invasion, apoptosis, proliferation and cancer stem cells were abolished in β-catenin overexpressing cells (figure 3*c–g*). And this was further confirmed using the freshly isolated NSCLC cells (electronic supplementary material, figure S2). Taken together, these results suggest that IL-38 may inhibit NSCLC cells via the β-catenin pathway.

**Figure 3.** IL-38 inhibits β-catenin expression in NSCLC cells. (*a*) The mRNA level of β-catenin was measured by qPCR. A549 and SK-MES-1 cells were treated with 100 ng ml^−1^ rhIL-38. *n* = 3. *p < 0.05. (*b*) The protein level of β-catenin was measured by western blot. A549 and SK-MES-1 cells were treated with 100 ng ml^−1^ rhIL-38. *n* = 3. *p < 0.05. (*c*–*g*) The wound healing, cell invasion, apoptosis and survival rates and the clone-forming ability of cells overexpressing β-catenin or empty vector were analysed. Cells were treated with 100 ng ml^−1^ rhIL-38. *n* = 3. *p < 0.05.

### 3.4. Overexpression of IL-38 suppresses non-small cell lung cancer development *in vivo* and increases the sensitivity to chemotherapeutic drugs

To investigate the role of IL-38 in tumourigenesis, a xenograft NSCLC model was used. The SK-MES-1 cells were cultured, collected and injected into mice. After each tumour reached macroscopic size, pAAV-IL38 was administered by intravenous injection weekly for 4 weeks. The IL-38 therapy could suppress the tumour growth significantly (figure 4*a*,*b*). Tumour cells were isolated from the mice and then subjected to chemotherapeutic drugs. Data showed that IL-38 treatment sensitized the NSCLC to the drugs 5-fluorouracil, cisplatin and doxorubicin. These results suggest that IL-38 plays a vital role in suppressing tumourigenicity *in vivo* and might sensitize the tumours to chemotherapy.

**Figure 4.** IL-38 suppresses NSCLC tumourigenesis *in vivo*. The adeno-associated virus expressing IL-38 or GFP was administered via tail-vein injection. The average tumour weight (*a*) and the tumour size (*b*) were analysed. Tumour cells were isolated from the mice and then subjected to chemotherapeutic drug treatment (*c*)*. n* = 12. *p < 0.05.

## 4. Discussion

Lung cancer is one of the most common malignancies worldwide, and it remains the leading cause of cancer-related death with low early-stage diagnosis rate. Owing to the complexity and heterogeneity of this disease, the early diagnosis of lung cancer can improve survival rate. Therefore, more efforts should be made to uncover the underlying mechanisms and develop novel therapeutic targets.

IL-38 has been identified as a natural suppressor of innate inflammatory and immune responses [7–9]. It is highly expressed in inflammatory tissues to inhibit the excessive inflammatory response. However, there is little information about how IL-38 influences the pathogenesis of NSCLC development, progression and prognosis. The function of IL-38 in tumours is largely unknown. Inflammation is the seventh hallmark of tumours [11], inferring that IL-38 might influence inflammation-related tumours. Here, we provided the evidence that IL-38 suppresses NSCLC progression through β-catenin suppression.

In the current study, we first investigated the expression pattern of IL-38 protein in NSCLC patients. We found that IL-38 was expressed in non-tumour tissues and it was downregulated in cancer tissues. Further analysis showed that the lack of IL-38 was tightly associated with cancer metastasis and poor survival, indicating that IL-38 could be developed as a novel prognostic marker to predict tumour recurrence.

To confirm our clinical findings, we treated NSCLC cell lines A549 and SK-MES-1 with different concentrations of IL-38. We found that IL-38 suppressed migration, invasion and cell growth of NSCLC cancer *in vitro*. In the meantime, IL-38 also promoted NSCLC apoptosis and reduced cancer stem cells. Aberrant activation of β-catenin contributes to NSCLC progression [10]. To gain further insight into the role of IL-38 in NSCLC, we examined the expression of β-catenin. We found that IL-38 downregulated the expression of β-catenin at both mRNA and protein level. In our study, the reduced expression of β-catenin may explain the anti-tumour and anti-proliferative activity of IL-38. Furthermore, we also confirmed the anti-tumour effects of IL-38 in a mouse model of NSCLC and demonstrated that IL-38 could sensitize the NSCLC to chemotherapeutic drugs.

Although several reports showed that IL-38 was highly expressed in lung cancer [12,13], our study here demonstrated that the downregulated expression of IL-38 in cancer tissues compared to the adjacent tissues was associated with NSCLC progression. The reason for the divergent results between our study and previous reports remains unclear. It might be the differences of study design or patient population. And this type of opposite function of an anti-inflammatory factor in tumour progression has also been demonstrated for IL-35 in hepatocellular carcinoma [14–16]. Thus the function of the anti-inflammatory factors in tumour progression might be complicated and further studies are necessary to uncover the anti-tumour mechanisms of IL-38 in NSCLC.

In conclusion, our data showed that IL-38 expression is lower in NSCLC. By inhibiting β-catenin expression, IL-38 impeded NSCLC development. Thus, IL-38 could be a potential candidate for immunotherapy in NSCLC. However, the manner in which IL-38 diminishes the expression of β-catenin in NSCLC is not clear.

## 5. Conclusion

Our results indicate that IL-38 is decreased in human NSCLC and IL-38 is capable of exerting anti-tumour activity by suppressing β-catenin expression. Our findings suggest that IL-38 may have clinical potential not only as a promising prognostic predictor to identify individuals with poor prognostic potential, but also as a novel therapeutic target in the treatment of NSCLC.

## Supplementary Material

Supplementary Fig 1

## Supplementary Material

Supplementary Fig 2

## Data accessibility

All data have been submitted as figures in the main text or electronic supplementary material.
